# The Present SP Tests for Determining the Transition Temperature T_SP_ on “U” Notch Disc Specimens

**DOI:** 10.3390/ma10050490

**Published:** 2017-05-03

**Authors:** Karel Matocha, Ondrej Dorazil, Roger Hurst

**Affiliations:** 1 Department of Material Engineering, Faculty of Metallurgy and Materials Engineering, VŠB—Technical University of Ostrava, 17. Liostopadu 2172/15, 708 00 Ostrava, Czech Republic; 2 MATERIAL & METALLURGICAL RESEARCH Ltd., Pohranicni 31, 703 00 Ostrava-Vitkovice, Czech Republic; ondrej.dorazil@mmvyzkum.cz; 3 Institute of Structural Materials, College of Engineering, Swansea University, Swansea SA2 8PP, UK; r.c.hurst@plnet.nl

**Keywords:** small punch testing, SP transition temperature T_SP_, notched disc specimen, plane disc specimen, impact energy, fracture appearance transition temperature (FATT), ductile brittle transition temperature (DBTT), transition temperature (TT)

## Abstract

The principal difference between the small punch (SP) testing technique and standardized impact testing lies in the fact that the SP tests carried out in accordance with CWA 15627 Small Punch Test Method for Metallic Materials use disc-shaped test specimens without a notch. Especially in tough materials, the temperature dependence of SP fracture energy E^SP^ in the transition area is very steep and lies close to the temperature of liquid nitrogen. In this case, the determination of SP transition temperature T_SP_ can lead to significant errors in its determination. Efforts to move the transition area of penetration testing closer to the transition area of standardized impact tests led to the proposal of the notched disc specimen 8 mm in diameter and 0.5 mm in thickness with a “U” shaped notch 0.2 mm deep in the axis plane of the disc. The paper summarizes the results obtained to date when determining the transition temperature of SP tests T_SP_, determined according to CWA 15627 for material of pipes made of P92, P22, and a heat treated 14MoV6-3 steel in the as delivered state. Although the results obtained confirmed the results of other works in that the presence of a notch in a SP disc is insufficient to increase the transition temperature significantly and certainly not to the values obtained by Charpy testing, comparison of the different behaviors of the alloys tested reveals some evidence that the notch reduces the energy for initiation. This implies that the test on a notched disc is more a test of crack growth and would be a useful instrument if included in the forthcoming EU standard for SP testing.

## 1. Introduction

CWA 15627 Part B: A Code of Practice for Small Punch Testing for Tensile and Fracture Behavior (“the Code”) describes the procedures recommended for determination of yield stress YS, ultimate tensile strength UTS, DBTT (measured by fracture appearance transition temperature (FATT) and/or absorbed energy transition temperature (TT) (for example 41J) and fracture toughness J_IC_ of the metallic materials from the results of SP tests [1,2].

DBTT expressed as FATT is correlated according to the Code with T_SP_ (SP transition temperature), determined from the results of SP tests in the temperature range −193 °C to +23 °C in the form [1,2,3,4]:

T_SP_ = *α* FATT_Charpy_ or FATT_Charpy_ = T_SP_*β* + A (1)

Typical values for *α* for structural steels have been reported to be around 0.35 [5,6] indicative of much lower transition temperatures realized during the SP test than with conventional Charpy methods. The SP transition temperature T_SP_ is determined according to the Code as the temperature where E^SP^ has its mean value of the highest and the lowest values in the transition region, by intersecting the smooth curve fitted from the energy versus temperature dependence of fracture energy E^SP^ [1]. The SP fracture energy E^SP^ is determined by integration of the force–displacement curve up to fracture [1]:

(2) $$E^{\mathrm{SP}}=\;\overset{u_{f}}{\underset{0}{\int }}F\left(u\right)du$$

where u*_f_* is defined according to Code as the punch displacement at 20% load drop after maximum load F_m_ (F_f_ = 0.8 . F_m_).

Multiple load drops are observed from time to time at load–punch displacement curve at the SP tests carried out at lower temperatures [4,7]. By monitoring the bulged surface of the disc during the SP test with a camera in author laboratory [8] it has been shown, that the occurrence of the first load drop is a consequence of the initiation of the first circumferential crack with the following load drop associated with the propagation of further radial cracks. In such cases, the SP fracture energy E^SP^ should be calculated as the area under the load–punch displacement curve up to first load drop. However, the determination of SP transition temperature T_SP_ in accordance with CWA 15627 and from energy for the initiation of the first crack was found to be insignificant [4,8].

The principal difference between the SP testing technique and standardized impact testing lies in the fact that the SP tests carried out in accordance with the Code use disc-shaped test specimens without a notch. Especially in tough materials, the temperature dependence of fracture energy in the transition area is very steep and lies close to the temperature of liquid nitrogen. The procedure recommended in the CWA for the determination of T_SP_ can, in this case, lead to significant errors in its determination [9]. Efforts to move the transition area of small punch testing closer to the transition area of standardized impact tests led to the proposal of the notched disc specimen. Up to the present, only very few authors have introduced a notch in small punch testing, mostly in relatively recent studies [9,10,11,12]. However, the introduction of a sharp circular notch with a notch tip radius <5 μm and of diameter equal to the punch diameter with the intention of maximizing the notch tip load equally around the notch circumference did not result in the displacement of SP transition temperature T_SP_ towards the FATT obtained from conventional Charpy V notch tests [13]. The most recent attempts in the authors’ laboratories to investigate the effect of notch geometry on SP transition temperature have used both scratched (an orthogonal cross of 50 μm [14]) and a diametral EDM notch 200 μm deep [15] on a disc removed from reactor pressure vessel steel. Although both types of notch contributed significantly to the initiation of the fracture process they were found to have little effect on the ductile brittle transition temperature, even with high strain rate testing closer to Charpy conditions. Nevertheless, it is under consideration to include notched disc testing in the proposed standard on SP testing and additional testing programs are required to enable this decision to be taken. For this reason, and based on the results from published efforts cited above, it has been decided to extend the study to additional materials but concentrating on the diametral 0.2 mm notched disc.

Figure 1 shows disc test specimen with a ‘‘U’’ shaped notch 0.2 mm deep in the axis plane of the disc [2,14].

The first results of SP tests at lower temperatures carried out on 14 MoV6-3 steel indicated that the use of the notched specimens could shift the transition temperature T_SP_ to higher temperatures to a limited extent but not to the much higher transition temperatures obtained using Charpy testing (Table 2 below). Beyond the maximum fracture energy, the temperature dependence of fracture energy was found also to be less steep (see Figure 2). 

In the present paper, these results will be compared with results obtained for tube ø 219 × 22.2 mm^2^ in as received state made of P92 steel and tube ø 508 × 25 mm^2^ in as received state made of P22 steel. 

## 2. Test Material

Table 1 summarizes the controlled chemical composition of the testing materials.

Table 2 summarizes the tensile behavior at ambient temperature using round bars 8 mm in diameter. Test specimens were oriented in longitudinal direction.

Microstructure of the P92 steel is composed of tempered martensite while microstructure of the P22 steel is tempered bainitic and the steel 14MoV6-3 is formed by mixture of tempered ferrite and bainite. Table 3 summarizes transition temperatures FATT and impact energies measured at FATT temperatures using Charpy V test specimens (KV)_FATT_ and Charpy U test specimens (KU)_FATT_ with notch 2 mm deep. All test specimens were oriented in tangential direction.

Although the P92 steel has approximately the same FATT temperature as the steels P22 and 14MoV6-3 the fracture initiation energy ((KU)_FATT_-(KV)_FATT_) of this steel is significantly lower.

## 3. Small Punch Test Results and Discussion

SP tests at −193 °C up to ambient temperature were carried out on the servo-mechanical testing machine Lab Test 5.10ST following the procedures set out in [1], under crosshead control at crosshead speed of 1.5 mm/min with puncher 2 mm in diameter using discs 8 mm in diameter and 0.5 ± 0.005 mm thickness. The load–cross head displacement curve was monitored during each SP test. 

Figure 3 and Figure 4 show the temperature dependences of the fracture energy E^SP^ determined for P22 steel and P92 steel respectively using both plane disc specimens and disc specimens with the 0.2 mm deep notch. It can clearly be seen in Figure 3 that the increase in the small punch transition temperature for the P22 steel as a result of the introduction of the notch, namely from 89 K to 105 K is very similar to the result for the 14MoV6-3 shown in Figure 2. Again, the increase in value falls very much below the transition temperature obtained from the conventional Charpy test (Table 3). Whereas the SP Fracture energy/ temperature curves for the un-notched 14M0V6-3 and P22 steels are almost identical, the notched P22 curve does not show a less steep dependence of fracture energy on temperature beyond the maximum energy, with the curve running in parallel to the un-notched results. A few repeat tests on the notched discs over the temperature range 90 to 130 K may clarify whether this minor difference between the P22 and 14MoV6-3 notched results is worthy of further investigation. 

The fracture results for the P92 steel (Figure 4) are quite different to those for the other two alloys. The T_SP_ of 146 K derived from the un-notched tests and the maximum fracture energy is reached around 170 K, the transition part of the curve being much less steep than for 14MoV6-3 and P22 but reaching higher temperatures. This higher value for the SP transition temperature compares with the value of 133 K reported by Blagoeva et al. [16] for the comparable alloy P91. In comparison with the two lower alloy steels, there is no shift in the curve observed for the notched test at low temperatures, where the curve appears to follow exactly the same rise in fracture energy with temperature until around 150 K, coincidentally around the T_SP_ for the un-notched test, where the fracture energy commences its fall with further increase in temperature. A similar lack of displacement of the notched curve was also reported for alloy P91 but for 1 mm thick discs with and without 0.5 mm deep notches by Turba et al. [13]. As a result of this lack of displacement of the curve to higher temperatures, the T_SP_ for the P92 notched test is characterized by the lower value of 124 K. In this case, the introduction of a notch played no role in increasing the SP transition temperature towards the Charpy value, in fact quite the reverse. 

For all these types of notched SP test, it is important to understand the role played by the initiation of the crack and the energy for crack growth. Although the presence of the notch will undoubtedly play a role in crack initiation the results show that the effect of the notch in the Charpy test is much more dominant, indicating that the main effect in the notched SP test lies with the crack propagation. As a result, the transition temperatures found in the notched tests are not so much affected by the notch but the fracture energies are certainly reduced for the notched specimens. This could simply be caused by the difference in ligament length, 0.5 mm for the un-notched and 0.3 mm for the notched, through which the crack must propagate. This is also apparent in the results for P91 [13] where the fracture energy for a 1 mm thick disc is clearly greater than for a 0.5 mm thick disc. We intend to investigate this aspect in future work by testing plain discs of 0.3 mm thickness and notched specimens with 0.1 mm deep notches along with plain specimens of 0.4 mm thickness.

Of considerable importance in the application of SP fracture testing is the acceptance of plant operators whether they can rely on the *α* values obtained in predicting the FATT or DBTT properties for components, in particular where degradation in long term properties may be expected for example through irradiation, creep, or other microstructural damage. As Table 4 shows the ratio of T_SP_/FATT determined using plane discs is significantly dependent on the type of material, although the differences appear to be less for the notched discs. For this reason, it would still appear to be justifiable to include notched SP tests in the forthcoming EN standard although a much more fundamental understanding of the actual role of the notch is required.

## 4. Conclusions

On the basis of temperature dependences of small punch fracture energy E^SP^ determined for P92, P22, and 14MoV6-3 steels with different microstructures using both plane and notched disc test specimens and impact tests for determination of FATT temperature it is possible to make the following conclusions:

(1) The introduction of a 0.2 mm U-shaped notch into a standard 0.5 mm SP disc specimen raises to a limited extent the measured ductile brittle transition temperature for P22 and 14MoV6-3 steels while marginally reducing the transition temperature for the P92 steel.
(2) This confirms the results of other workers looking at different sizes and shapes of notches and indeed different materials that it is not possible to raise the transition temperature using a notched SP disc to the levels measured in a conventional Charpy test.
(3) However, with increasing data being made available for the correlation of SP and Charpy fracture transition temperature using the relationship *α* = (T_SP_)_notch_/FATT, it is conceivable that the consistency of *α* values may be improved by obtaining them with notched SP tests and to this end these tests could usefully be introduced into the EN standard for SP testing presently in preparation.

## Figures and Tables

**Figure 1:** Disc test specimen with “U” notch in the axis of disc plane. (**a**) Figure of the disc specimen; (**b**) dimensions of the notch.

**Figure 2:** The effect of the notch on temperature dependence of fracture energy of penetration test. Pipe ø 457 × 28 mm^2^ made of 14MoV6-3 steel after heat treatment 940 °C/1 h/air + 720 °C/2 h/air. Crosshead speed 1.5 mm·min^−1^, punch diameter 2.0 mm (adapted from [2] with permission of publisher).

**Figure 3:** Temperature dependence of small punch transition temperature T_SP_ determined for P22 steel using plane disc specimens 0.5 mm in thickness and disc specimens with 0.2 mm deep notch.

**Figure 4:** Temperature dependence of small punch transition temperature T_SP_ determined for P92 steel using plane disc specimens 0.5 mm in thickness and disc specimens with 0.2 mm deep notch.

**Table 1:** The chemical composition of studied materials (weight %).

Material	C	Mn	Si	S	P	Cr	Mo	Ni	V
14MoV6-3	0.12	0.57	0.19	0.005	0.009	0.57	0.52	0.08	0.32
P92	0.13	0.53	0.25	0.009	0.011	8.53	0.44	0.13	0.19
P22	0.13	0.46	0.24	0.017	0.011	2.25	0.92	0.06	0.012

**Table 2:** Tensile behavior of testing material at ambient temperature.

Material	YS (Mpa)	UTS (Mpa)	A (%)	Z (%)
P92	669	805	21.5	65
P22	433	566	28.5	77
14MoV6-3	403	536	30.3	83

**Table 3:** Results of impact tests.

Material	FATT (°C)	(KV)_FATT_ (J)	(KU)_FATT_ (J)
P92	−3	62	89
P22	−1	74	136
14MoV6-3	−10	117	173

**Table 4:** Ratios T_SP_/FATT obtained using both plane and notched discs.

Material	(T_SP_)_plane_ [K]	*α* = (T_SP_)_plane_/FATT	(T_SP_)_notch_ [K]	Α = (T_SP_)_notch_/FATT
P92	146	0.54	124	0.46
P22	89	0.33	105	0.39
14MoV6-3	94	0.40	113	0.43
